# Personalized Recommendation Algorithm for Movie Data Combining Rating Matrix and User Subjective Preference

**DOI:** 10.1155/2022/2970514

**Published:** 2022-08-09

**Authors:** Chang Liu

**Affiliations:** Zhewen Pictures Group Co.,Ltd, Hangzhou 31000, China

## Abstract

The film industry has also caught the fast train of Internet development. Various movie resources have come into view. Users need to spend a lot of time searching for movies they are interested in. This method wastes time and is very bad. The article proposes an NMF personalized movie recommendation algorithm, which can recommend movies to users based on their historical behavior and preference. The research results of the article show the following: (1) the experiment counts movie reviews of different users in the same time span. The results show that 48.42% of users have only commented on a movie once, 79.76% of users have posted less than or equal to 5 comments, and 89.92% of user reviews have posted less than or equal to 10 times. (2) In the comparative experiments of the NMF algorithm in different dimensions, the effect of the NMF-E algorithm is much better than that of the NMF-A algorithm. The accuracy, recall, and *F*1 value of the NME-E algorithm are all 3 types. The experimental results show that the NME-E algorithm is the best among all algorithms. (3) In the experiment to test the effectiveness of the NMF personalized recommendation algorithm, comparing the experimental results, the MAE value of the improved NMF personalized recommendation algorithm is lower than that of the unimproved algorithm. When the number of neighbors is 10, the highest value of the improved MAE of the previous algorithm is 0.837. After the improved algorithm, the MAE value is the highest (0.83), and the MAE value has dropped by 0.007, indicating that the error is smaller after the improved algorithm, and the result of recommending movies is more accurate. The recall value of the four algorithms will increase as the number of neighbors increases. Among them, the recall value of the NMF algorithm proposed in the article is the highest among several algorithms. The highest value can reach 0.200, which is higher than the highest value of other algorithms. It shows that the recommendation effect of NMF algorithm is the best. (4) According to the results of the questionnaire, after using the NMF personalized recommendation algorithm, users' satisfaction increased from 20% to 50%, an increase of 30%, and their dissatisfaction decreased from 15% to 8%, a decrease of 7%. Relative satisfaction increased from 52% to 55%, an increase of 3%, satisfaction increased from 35% to 60%, an increase of 25%, and dissatisfaction decreased from 40% to 20%, a decrease of 20%, indicating that the algorithm can meet the requirements of most people.

## 1. Introduction

With the rapid development of the information age, we will be faced with very complex digital and networked data. How users choose effective information from the tedious information, personalized recommendation algorithms can help users filter out the information they want and solve the needs of the vast majority of people. The film industry in China has also been developing rapidly in recent years. There are many movies released every year. The personalized recommendation of movie data can effectively solve the different needs of users. There are many types of movies released every year in our country. When faced with so many movies, users will inevitably be at a loss and do not know how to choose. Literature [1] proposed a new cross-space affinity learning algorithm on different spaces with heterogeneous structures. The algorithm records and saves the record of the movie watched by the user, as well as the record of the comment. According to the user's comment, the user's movie hobby can be calculated. The article also compares the performance of the algorithm with the benchmark movie recommendation set, and the results show that the algorithm proposed in the article has advantages. Literature [2] focuses on how to design a reliable and highly accurate movie recommendation algorithm. Literature [3] proposed an improved deep reinforcement learning algorithm to recommend movies. Literature [4] proposed an efficient privacy protection collaborative filtering algorithm based on differential privacy protection and time factors. Literature [5] discussed the problems of traditional collaborative filtering algorithms and proposed improvements. Literature [6] introduced virtual prediction items in a relatively sparse rating database. Literature [7] is combining collaborative filtering and association rules to accurately improve user recommendations. Literature [8] proposed a hybrid collaborative filtering algorithm based on user preferences and item characteristics. Literature [9] is inspired by the user-item rating matrix of the network and introduces an improved algorithm that combines the similarity of items with the dynamic resource allocation process. Aiming at the problem of insufficient demand mining for movie recommendation systems, literature [10] proposed a personalized movie recommendation system based on the collaborative filtering algorithm. Literature [11] proposed a spark-based matrix factorization recommendation algorithm, which uses spark memory computing and parallel data processing. Literature [12] focuses on the application of the latent factor model in the movie recommendation system and improves the latent factor model to overcome its shortcomings that it cannot give recommendation explanation. Literature [13] proposed a distributed collaborative filtering recommendation algorithm. Literature [14] researched using the concept of data warehouse to create a movie recommendation system. Literature [15] introduced the theory of semantic computing to label the semantic tags in movie clips and candidate advertisements.

## 2. Research on Personalized Movie Recommendation Technology

### 2.1. Research Background and Significance

This paper considers the introduction of other important movie information under the framework of collaborative filtering algorithm and combined with scoring data for hybrid recommendation [16]. It is worth noting that there is a kind of rich and valuable information on movie websites-movie reviews, but this kind of information is often ignored. Movie sites do hope that users can give more and more detailed reviews because considering that when users decide whether to watch a movie, the movie reviews given by other users will provide them with reference opinions, and a large number of movie reviews can improve users' perceptions. The level of interaction between users, thereby, potentially increases user stickiness. Generally, users always express the points or aspects that they care about most in their reviews of a certain movie, and these aspects often reflect the user's potential preference for the movie. A general rating can only indicate whether a user likes the movie or not, but it cannot give a specific reason why the user likes or hates the movie [17]. The user's specific evaluation of the movie is shown in Table 1.

### 2.2. Current Status of Movie Recommendation Research

Since review information is user-generated content, which contains the opinions and emotions of the reviewer, it is worth digging deeper to describe the “unique attributes” of users by using the review text. However, in the field of movie recommendation, film reviews should be digging. Relatively speaking, there are still very few studies. From the perspective of the recommendation field as a whole, some researchers have realized the rich information contained in text reviews and the value contained therein, but most of the researches use topic models to directly extract the topic distribution of text reviews without considering to the emotional factor in the comments. The user's film reviews actually reflect the user's likes and dislikes of a movie from certain angles. The previous research mixed texts with different emotional tendencies for analysis and could not fully extract the user's favorite and dissatisfied aspects of the movie. The use of sentiment analysis is to refine and divide the reviews and extract the user's satisfaction and dissatisfaction with the movie, which is the significance of mining reviews [18].

### 2.3. Personalized Recommendation Process

It can be regarded as first data collection of movie information evaluated by users, combined with user's movie reviews for sentiment analysis, and then imported into the NMF personalized recommendation model. The model will predict the movies that the user may like based on the user's historical behavior information and the supervisor's preference. Sort the movies according to the degree of preference. The first one is the one that the user may be most interested in, and then the list is recommended to the user. The basic flow chart is shown in Figure 1.

## 3. Research on the Recommendation Algorithm of Scoring Matrix and User Supervisor Preference

### 3.1. User Subjective Preference Recommendation Algorithm

The recommended algorithm steps are shown in Figure 2.

Construct a user movie rating table, as shown in Table 2.

*I*_*u*_ is a collection of movies rated by user *u*, and *I*_*v*_ is a collection of movies rated by user *v* [19]; user similarity is

(1) $$\begin{array}{c} \text{sim}\left(u,v\right)\frac{\left|I_{u}\cap I_{v}\right|}{\left|I_{u}\cup I_{v}\right|}. \end{array}$$

Recommended results:

(2) $$\begin{array}{c} {\bar{r}}_{ui}=\sum_{j\in S\left(j,k\right)\cap N\left(u\right)}\text{sim}\left(i,j\right)r_{ui}. \end{array}$$

*N*(*u*) is a collection of movies rated by the user *u*, and *S*(*j*, *k*) is a collection of movies *j* similar to K movie collections [20].

The formula for calculating the degree of preference between user *u* and other movies *v* is

(3) $$\begin{array}{c} S\left(u,v\right)=\sum_{V\in N\left(u\right)}\cos\left(R{\left(:,v\right)}^{T},R\left(:,v\right)\right). \end{array}$$

Common mixed recommendation models are shown in Table 3:

Build user characteristics such as in Table 4.

Calculate user *G*'s preference for your teenage movie:

(4) $$\begin{array}{c} r=\frac{1}{n}\sum_{i=1}^{n}\left(x_{i}-\text{ave}\right). \end{array}$$

Movies users may like

(5) $$\begin{array}{c} \cos\left(U,I\right)=\frac{\sum U_{a}\times I_{a}}{\sqrt{\sum U_{a}^{2}\times \sqrt{\sum I_{a}^{2}}}}. \end{array}$$

Error value of movie prediction:

(6) $$\begin{array}{c} \text{MAE}=\frac{\sum_{u,i\in T}\left|r_{ui}-{\bar{r}}_{ui}\right|}{N}. \end{array}$$

Movie recommendation accuracy rate:

(7) $$\begin{array}{c} \text{RMSE}=\frac{\sqrt{\sum_{u,i\in T}{\left(r_{ui}-{\bar{r}}_{ui}\right)}^{2}}}{N}. \end{array}$$

Movie ranking prediction:

(8) $$\begin{array}{c} \text{Precision}=\frac{\sum_{u\in U}\left|R\left(u\right)\cap T\left(u\right)\right|}{\sum_{u\in U}\left|R\left(u\right)\right|}. \end{array}$$

### 3.2. Score Matrix Recommendation Algorithm

In the recommendation system, *U*^*m*^={*u*_1_, *u*_2_,…, *u*_*m*_} represents the user level, *I*^*n*^={*i*_1_, *i*_2_,…, *i*_*n*_} represents the movie set, and *R*^*mn*^ represents the *m* × *n*-dimensional rating matrix [21] as shown in Table 5.

The similarity between users is expressed as

(9) $$\begin{array}{c} \text{PCC}\_\text{sim}\left(a,b\right)=\frac{\sum_{p\in P}\left(r_{a,p}-{\bar{r}}_{a,p}\right)\left(r_{b,p}-{\bar{r}}_{b,p}\right)}{\sqrt{\sum_{p\in P}\left(r_{a,p}-{\bar{r}}_{a,p}\right)\sqrt{\sum_{p\in P}\left(r_{b,p}-{\bar{r}}_{b,p}\right)}}}. \end{array}$$

Among them, *P* represents the collection of movies that users *a* and *b* have rated together, and ${\bar{r}}_{a,p}$ and ${\bar{r}}_{b,p}$ represent the average ratings of users and based on the common movie collection *P*, respectively.

Cosine similarity:

(10) $$\begin{array}{c} \mathrm{Cos}\;\_\text{sim}\left(a,b\right)=\frac{\overset{⟶}{a}\cdot \overset{⟶}{b}}{\left|\overset{⟶}{a}\right|*\left|\overset{⟶}{b}\right|}. \end{array}$$

The formula can also be written as

(11) $$\begin{array}{c} \text{Cos}\_\text{sim}\left(a,b\right)=\frac{\sum_{p\in P}r_{a,p}*r_{b,p}}{\sqrt{\sum_{p\in P}r_{a,p}^{2}}\sqrt{\sum_{p\in P}r_{b,p}^{2}}}. \end{array}$$

Select the first *K* similar users to rate the unreviewed movie collection [22]; the calculation formula is

(12) $$\begin{array}{c} \text{pre}\left(a,p\right)={\bar{r}}_{a}+\frac{\sum_{b\in NN}\text{sim}\left(a,b\right)*\left(r_{b,p}-{\bar{r}}_{b}\right)}{\sum_{b\in NN}\text{sim}\left(a,b\right)}. \end{array}$$

User *u*'s rating calculation formula for unrated movie *p*:

(13) $$\begin{array}{c} \text{pre}\left(u,p\right)=\frac{\sum_{i\in NN}\text{sim}\left(i,p\right)*r_{u,i}}{\sum_{i\in NN}\text{sim}\left(i,p\right)}. \end{array}$$

### 3.3. NMF Personalized Recommendation Algorithm

The NMF personalized recommendation algorithm combining the scoring matrix and the user's subjective preference is to extract and generate each user's comment [23] and calculate the weight, as shown in Table 6:

${\bar{r}}_{i}$ Is the average rating of user *u*_*i*_ on the movie.

Calculate the interest topics of a user's single movie review:

(14) $$\begin{array}{c} \theta_{ij}=\alpha_{p}\cdot \theta_{p-i,j}+\alpha_{N}\cdot \theta_{N-i,j}. \end{array}$$

The formula for calculating the overall interest distribution of users is

(15) $$\begin{array}{c} \theta_{i}=\frac{\sum_{j\in I_{i}\theta_{ij}}}{\left|I_{i}\right|}. \end{array}$$

The following formula measures the similarity between users:

(16) $$\begin{array}{c} D_{KL}\left(\theta_{a}\|\theta_{b}\right)=\sum_{i}\theta_{a}\left(i\right)\ln\frac{\theta_{a}\left(i\right)}{\theta_{b}\left(i\right)},\\ \overset{⟶}{M}=\frac{1}{2}\left(\theta_{a}+\theta_{b}\right),\\ D_{JS}\left(\theta_{a}\|\theta_{b}\right)=\frac{1}{2}\left(D_{KL}\left(\theta_{a}\|\overset{⟶}{M}\right)+D_{KL}\left(\theta_{b}\|\overset{⟶}{M}\right)\right),\\ \text{sim}\left(a,b\right)=1-D_{JS}\left(\theta_{a}\|\overset{⟶}{M}\right). \end{array}$$

Average the topic distribution of all film reviews:

(17) $$\begin{array}{c} \theta_{j}=\frac{\sum_{i\in U_{j}\theta_{ij}}}{\left|U_{j}\right|}. \end{array}$$

Predict the distance between the user and the movie according to *U*, *V*:

(18) $$\begin{array}{c} U_{u}=U_{u}-\alpha \frac{\partial L}{\partial U_{u}},\\ V_{i}=V_{i}-\alpha \frac{\partial L}{\partial V_{i}},\\ b_{u}\left(u\right)=b_{u}\left(u\right)-\alpha \frac{\partial L}{\partial b_{u}\left(u\right)},\\ b_{i}\left(i\right)=b_{i}\left(i\right)-\alpha \frac{\partial L}{\partial b_{i}\left(i\right)}, \end{array}$$

in

(19) $$\begin{array}{c} \frac{\partial L}{\partial U_{u}}=-\sum_{i=1}^{n}I_{ui}T_{ui}\left(Y_{ui}-{\bar{\text{d}}}_{ui}\right)\times \frac{1}{D_{ui}}\left(U_{u}-V_{i}\right)+\lambda U_{u},\\ \frac{\partial L}{\partial U_{i}}=-\sum_{u=1}^{m}I_{ui}T_{ui}\left(Y_{ui}-{\bar{\text{d}}}_{ui}\right)\times \frac{-1}{D_{ui}}\left(U_{u}-V_{i}\right)+\lambda U_{i},\\ \frac{\partial L}{\partial b_{u}\left(i\right)}=-\sum_{i=1}^{n}I_{ui}T_{ui}\left(Y_{ui}-{\bar{\text{d}}}_{ui}\right)+\lambda b_{u}\left(i\right),\\ \frac{\partial L}{\partial b_{i}\left(u\right)}=-\sum_{u=1}^{m}I_{ui}T_{ui}\left(Y_{ui}-{\bar{\text{d}}}_{ui}\right)+\lambda b_{i}\left(u\right). \end{array}$$

## 4. Simulation Experiment

### 4.1. Data Set Characteristics

The experiment selected a real user evaluation album with a time span of 2016.9.1–2017.1.14. The experiment recorded the ID of each user, the content and value of the rating, and the time of the rating. The experiment was carried out on each user who scored. Statistics on the total number of comments has been made. The results show that 48.42% of users have only commented on the movie once, 79.76% of users have commented less than or equal to 5 times, and 89.92% of users have commented less than or equal to 10 times. The results are shown in Tables 7 and 8.

### 4.2. Evaluation Criteria

The evaluation criteria are shown in Table 9.

### 4.3. Experimental Results and Analysis

The experiment compares the NMF personalized recommendation algorithm in different dimensions to verify the rationality and performance superiority of the algorithm. An algorithm in the experiment is to only collect user movie reviews without any analysis. This algorithm is called NMF-E for short. The second algorithm ignores the influence of some negative reviews in movie reviews on user interest topics, and only considers positive movie reviews. This algorithm is referred to as NMF-A for short. The experimental comparison results are shown in Figures 3–5:

According to the results of the comparative experiment, we can find that the NMF-E algorithm, which does not do any sentiment analysis on the movie reviews posted by users, is better than ignoring the impact of some negative reviews in movie reviews on user interest topics and only takes into account the positive reviews. The effect of the NMF-A algorithm of the movie review is much better. The accuracy, recall, and *F*1 value of the NME-E algorithm are the highest among the three algorithms. The accuracy and *F*1 value will decrease as the number of movies recommended by the user increases, and the recall rate will follow the user recommendation. The number of movies decreases as the number of movies increases.

### 4.4. Model Performance Testing

In order to test the effectiveness of the NMF personalized recommendation algorithm, we selected more than 100,000 comments on more than 1,000 movies from more than 900 users, and each user has more than 20 comments on the movie. In order to improve the accuracy of the NMF algorithm and find the most suitable decomposition dimension value, we can conclude from the data in the graph that the value of MAE will first decrease and then increase as the decomposition dimension increases. When the decomposition dimension value is at 6 o'clock, the value of MAE is the lowest. The value of MAE represents the accuracy of the algorithm for personalized recommendation of movies according to the user's preferences, and the recall value is reflected in the recommended movie results, the proportion of users who are really interested in the movie [24]. Among them, the value of MAE is small, indicating that the error of the algorithm is lower, and the value of recall is larger, indicating that the proportion of users who are really interested is more. The relationship between the decomposition dimension and MAE is shown in Figure 6.

After improving the NMF personalized recommendation algorithm, we compare it with the traditional NMF algorithm. Under the condition that the adjacent numbers of the variables are set to 10, 20, 30, 40, and 50, respectively, we compare the MAE values of the two different algorithms. The experimental data is shown in Figure 7:

From the data in the figure, we can conclude that the MAE value of the improved NMF personalized recommendation algorithm is lower than that of the unimproved algorithm. When the number of neighbors is 10, the highest MAE value of the algorithm before the improvement is 0.837. After the algorithm is improved, the MAE value is the highest value is 0.83, and the MAE value has dropped by 0.007, indicating that the error is smaller after the improved algorithm, and the result of recommending movies is more accurate. In order to further test the effectiveness of the NME algorithm, we compared with 3 other different algorithms and observed their MAE value and recall value. The details are shown in Tables 10 and 11.

From the data in Figure 8, we can conclude that the MAE values of the four algorithms will change with the fluctuation of the number of neighbors. When the number of neighbors is small, the MAE value of the NMF algorithm and the Jaccard algorithm fluctuates greatly. The NMF personalized recommendation algorithm proposed in the article among the four algorithms has the smallest MAE value regardless of the number of neighbors. When the number of neighbors is 10, the MAE value is the largest, and the maximum value is 0.783. The MAE value of the CEHPI algorithm is the largest among the four algorithms. The NCF and Jaccard algorithms are between the two algorithms. The experimental data further shows that the prediction accuracy of the NMF personalized recommendation algorithm proposed in the article is the highest among the four algorithms.

According to the data in Figure 9 and Table 11, we can conclude that the recall value of the four algorithms will increase as the number of neighbors increases. The recall value of the NMF algorithm proposed in the article is the highest among several algorithms, and the highest value can reach 0.200, both high and the highest value of other algorithms. The recall value of the Jaccard algorithm is the lowest among several algorithms, the lowest value is 0.100, and the CEHPI and NCF algorithms are somewhere in between.

### 4.5. Satisfaction Survey of Recommendation Results

In order to study the user's satisfaction after using the NMF personalized recommendation algorithm, the experiment took the form of questionnaire. The specific data is shown in Figure 10:

According to the data in Figure 10, after using the NMF personalized recommendation algorithm, the user's degree of satisfaction increased from 20% to 50%, an increase of 30%, and the degree of dissatisfaction decreased from 15% to 8%, a decrease of 7%. Relative satisfaction increased from 52% to 55%, an increase of 3%, satisfaction increased from 35% to 60%, an increase of 25%, and dissatisfaction decreased from 40% to 20%, a decrease of 20%. The experimental results prove that the NMF personalized recommendation algorithm can provide users with effective decision support, improve user satisfaction, and promote the long-term development of the film industry.

## 5. Conclusion

Movie reviews are important information that directly reflects the subjective feelings of users. According to user reviews, we can know the theme of the movie and the user's viewing experience. The article combines the scoring matrix and the personalized recommendation algorithm of movie data preferred by the user's supervisor and proposes an NMF personalized recommendation model. When users are faced with dazzling movie data, users no longer have to spend a lot of time searching for movies they are interested in. While the system meets the diverse needs of users, it also promotes the long-term development of the film industry [25]. According to the effective survey results, there are still some users whose satisfaction with the personalized recommendation model needs to be improved. Therefore, the performance of the personalized recommendation model should be continuously improved. This is the invincibility of the Chinese film industry in the face of increasing business competition.

## Figures and Tables

**Figure 1:** Flowchart of personalized recommendation.

**Figure 2:** Overview of user recommendation algorithm.

**Figure 3:** Accuracy curve.

**Figure 4:** Recall rate curve.

**Figure 5:** *F*1 measurement value curve.

**Figure 6:** Relationship between decomposition dimension and MAE value.

**Figure 7:** Improved algorithm performance comparison chart.

**Figure 8:** MAE values of different algorithms.

**Figure 9:** Recall values of algorithms.

**Figure 10:** User satisfaction survey.

**Table 1:** User evaluation form.

User ID	Time	Comment	score

68547261 (A)	2018-02-23 17:47:06	Watching “Interstellar,” the initial surprise comes from music. The first climax of the film is the appearance of the song called comfield chase. Perhaps the reason why this song became the core of the film is this kind of senseless spirit of exploration. Director Nolan said after listening to this piece: My movie is ready for shooting. Hans Zimmer's soundtrack makes this film the uncrowned king in many people's hearts.	4

58691048 (B)	2019-02-12 23:55:04	Why can this science fiction movie stand out and be included in the history of film and television? Interstellar is a real hard science fiction movie. The movie incorporates the concept of five-dimensional space. This is a film that fully uses the concept of time and space. Its script is more based on data theories and formulas to support the development of the entire plot. Compared with other movies with no scientific basis, it is judged high.	5

78651562 (C)	2018-10-25 9:53:09	“Interstellar,” Nolan is another magical film, and it should be the greatest science fiction film. Leaving aside the science fiction elements in the movie, after all, I do not understand [covering face]. From a human point of view, Nolan always likes to put the complexity of human nature in front of people, facing the instinct to survive, calling him the Earth. The hopeful professor Mann has become another Harvey Dante, with a feeling of DK series.	5

78961310 (D)	2014-11-16 00:49:28	Anne Hathaway said, I love him, but that does not mean I'm wrong. Love is something that humans cannot understand. It may be given to us by more advanced creatures. Although we think it is sensibility, it may be the highest level of wisdom. Anne Hathaway's short hair is very beautiful, like a smart and stubborn little boy, with human wisdom and love, who would not love her?	4

**Table 2:** User rating matrix.

User	Movie A	Movie B	Movie C	Movie D	Movie E

A	3	4	0	3.5	0
B	4	0	4.5	0	3.5
C	0	3.5	0	0	3
D	0	4	0	3.5	3

**Table 3:** Common mixed recommendation models.

Mixed way	Description

Weighted	The calculation results of multiple recommendation techniques are weighted and mixed to generate recommendations

Switching	The calculation results of multiple recommendation techniques are weighted and mixed to generate recommendations

Cascade	The cascading technology constructs the order of preference between different projects in the iterative refinement process

Combined	At the same time, multiple recommendation techniques are used to give multiple recommendation results to provide users with reference

Feature combination	The features generated by a specific recommendation technique are input to another recommendation technique

Increasing features	The output of the former recommended method is used as the input of the latter recommended method

Meta-level mixing	An internal model generated by one recommendation technique is used as an input for another recommendation technique

**Table 4:** User rating matrix.

User	Young you	Wolf warriors 2	Me and my motherland

User F	3	4	5
User G	—	3	6

**Table 5:** User-movie collection rating matrix.

User-movie collection	*i*_1_	*i*_2_	⋯	*i*_*j*_	⋯	*i*_*n*_

*u*_1_	*r*_11_	*r*_12_	⋯	*r*_1*j*_	⋯	*r*_1*n*_
*u*_2_	*r*_21_	*r*_22_	⋯	*r*_2*j*_	⋯	*r*_2*n*_
⋯	⋯	⋯	⋯	⋯	⋯	⋯
*u*_*i*_	*r*_*i*1_	*r*_*i*2_		*r*_*ij*_		*r*_*in*_
⋯	⋯	⋯	⋯	⋯	⋯	⋯
*u*_*m*_	*r*_*m*1_	*r*_*m*2_	⋯	*r*_*mj*_	⋯	*r*_*mn*_

**Table 6:** Weights of topic vectors.

	High score $\left(r_{ij}>{\bar{r}}_{i}\right)$	Low score $\left(r_{ij}>{\bar{r}}_{i}\right)$

Forward document weight	$\alpha_{p}=1/1+e^{-\left(r_{ij}>{\bar{r}}_{i}\right)}$	$\alpha_{p}=1/1+e^{r_{ij}-{\bar{r}}_{i}}$
Negative document weight	$\alpha_{N}=1/1+e^{r_{ij}-{\bar{r}}_{i}}$	$\alpha_{N}=1/1+e^{-\left(r_{ij}>{\bar{r}}_{i}\right)}$

**Table 7:** Evaluation record template.

User ID	Time	Movie IDmmc1	Score	Comment

61719620	2016-01-14 13:41:34	10577869	5	Love movie I really like! we met in the dark, of course we love each other, family feelings, family trivial matters, everything is so beautiful... Remember the English accent? The hostess is so beautiful! male starring in sunglasses, handsome! It's worth watching again anyway

**Table 8:** Statistics of user evaluation times.

Number of comments	User number	Percentage (%)

1	237209	48.42
≤5	390775	79.76
≤10	440539	89.92

**Table 9:** Evaluation criteria table.

	Metrics	Formula

Accuracy	The accuracy measurement standard refers to the ratio of the number of hit movies to the number of recommended movies. The larger the index value, the more accurate the recommendation result.	Precision=hits_*u*_/recset_*u*_

Recall rate	The recall rate standard refers to the ratio of the number of hit movies to the theoretical maximum number of hits. The larger the index value, the more accurate the recommendation result.	Recall=hits_*u*_/testset_*u*_

*F*1 measurement	The *F*1 measurement index can effectively balance the accuracy rate and the recall rate by favoring the smaller value. The larger the index value, the more accurate the recommendation result.	*F*1=2 × precision × recall/precision+recall

**Table 10:** MAE values of different algorithms.

Algorithm	5	10	15	20	25	30	35	40	45	50

NMF personalized recommendation algorithm	0.762	0.783	0.770	0.771	0.772	0.774	0.775	0.775	0.776	0.776
Jaccard personalized recommendation algorithm	0.815	0.790	0.790	0.791	0.795	0.797	0.802	0.803	0.804	0.809
CEHPI personalized recommendation algorithm	0.837	0.820	0.819	0.816	0.810	0.806	0.800	0.799	0.796	0.795
NCF personalized recommendation algorithm	0.810	0.791	0.790	0.790	0.785	0.784	0.783	0.782	0.780	0.779

**Table 11:** Recall values of different algorithms.

Algorithm	5	10	15	20	25	30	35	40	45	50

NMF personalized recommendation algorithm	0.042	0.058	0.100	0.130	0.157	0.184	0.185	0.188	0.776	0.200
Jaccard personalized recommendation algorithm	0.024	0.030	0.042	0.051	0.063	0.080	0.090	0.095	0.804	0.100
CEHPI personalized recommendation algorithm	0.024	0.031	0.051	0.060	0.073	0.110	0.115	0.117	0.796	0.120
NCF personalized recommendation algorithm	0.030	0.050	0.073	0.091	0.120	0.160	0.172	0.176	0.780	0.190

## Data Availability

The data used to support the findings of this study are available from the corresponding author upon request.
